# Microscopic Tumour Classification by Digital Mammography

This article has been retracted.

**DOI:** 10.1155/2021/6635947

**Published:** 2021-02-04

**Authors:** Jingjing Yang, Huichao Li, Ning Shi, Qifan Zhang, Yanan Liu

**Affiliations:** ^1^Affiliated Hospital of Hebei University, Baoding, Hebei 071000, China; ^2^School of Medical Technology, Qiqihar Medical College, Heilongjiang, Qiqihar 161006, China

## Abstract

In this paper, we investigate the classification of microscopic tumours using full digital mammography images. Firstly, to address the shortcomings of traditional image segmentation methods, two different deep learning methods are designed to achieve the segmentation of uterine fibroids. The deep lab model is used to optimize the lesion edge detailed information by using the void convolution algorithm and fully connected CRF, and the two semantic segmentation networks are compared to obtain the best results. The Mask RCNN case segmentation model is used to effectively extract features through the ResNet structure, combined with the RPN network to achieve effective use and fusion of features, and continuously optimize the network training to achieve a fine segmentation of the lesion area, and demonstrate the accuracy and feasibility of the two models in medical image segmentation. Histopathology was used to obtain ER, PR, HER scores, and Ki-67 percentage values for all patients. The Kaplan-Meier method was used for survival estimation, the Log-rank test was used for single-factor analysis, and Cox proportional risk regression was used for multifactor analysis. The prognostic value of each factor was calculated, as well as the factors affecting progression-free survival. This study was done to compare the imaging characteristics and diagnostic value of mammography and colour Doppler ultrasonography in nonspecific mastitis, improve the understanding of the imaging characteristics of nonspecific mastitis in these two examinations, improve the accuracy of the diagnosis of this type of disease, improve the ability of distinguishing it from breast cancer, and reduce the rate of misdiagnosis.

## 1. Introduction

A nonspecific mastitis is a group of chronic inflammatory diseases of the breast that do not occur during lactation and are not associated with bacterial infections [1]. Because of the atypical clinical symptoms, it is easy to be misdiagnosed as breast cancer; the imaging manifestations are complex and variable, lacking in specificity, and most difficult to distinguish from breast cancer [2]. Mammography, ultrasound, and MRI have their advantages in the diagnosis and differential diagnosis of nonspecific breast cancer, but each has certain limitations [3]. This article reviews the imaging characteristics of the main pathological types of nonspecific mastitis and the differential diagnosis [4]. Mammography is the most basic and commonly used method for diagnosing breast disease, with a sensitivity of 69%–90%. Foci of plasmatic mastitis are mainly located in the periareolar and subareolar regions, with different stages of pathology and different radiographic appearances [5]. Wu divided the X-ray manifestations of PCM into four types: inflammatory type, ductal dilatation type, local infiltration type, and nodular mass type and considered that the more valuable signs of X-rays for plasmatic mastitis are mainly asymmetric density increasing along the long axis of the ducts, with an uneven density of the foci, which may be accompanied by cystic, honeycomb, or ductal structure hypodensities, with scattered rods or small hollow spaces [6]. PCM is classified into acute, subacute, and chronic phases according to the clinical duration of the disease, and different clinical stages of PCM have different X-ray manifestations [7]. Deep learning is a branch of artificial intelligence that has demonstrated good performance in a variety of complex tasks, especially those related to images [8]. The field of medical imaging relies heavily on images to extract useful information, so it is one of the areas where deep learning has been applied most effectively, and research in this area has developed rapidly in recent years [9]. In this paper, we review the research progress of deep learning in medical imaging and discuss the opportunities and challenges of incorporating deep learning into future medical imaging [10]. The deep learning method based on convolutional neural networks has won an overwhelming victory in the ImageNet International Liquid Scale Visual Recognition Challenge (ILSVRC), and, for the first time, the error rate of the deep learning method is lower than that of human observation. Acquisition error rate: since then, the performance of deep learning algorithms for image classification has been improving and impressive results have been achieved in other areas [11]. Medical imaging differs from other aspects of medicine in that almost all the primary data and reports used for imaging are digital and these data are suitable for analysis by deep learning algorithms [12]. The potential applications of deep learning in medical imaging have become evident, and, in this paper, we will outline the applications of deep learning in medical imaging [13].

With sufficient data available, a deep neural network can be trained from scratch [14]. The size of the trained network model depends on the task and data characteristics [15]. However, common architectures used in medical imaging are based on AlexNet and VGG, which have fewer network layers and weights, and Wang et al. used a scratch-trained model for assessing the presence of Alzheimer's disease in cranial MRI-based deep learning [16]. Deeper network models include deep residual networks (ResNet) and the inception architecture, which are better applied to medical imaging [17]. Three different ResNets were applied to predict brain tumour MGMT methylation status in preoperative MRI with 94.9% accuracy, which is better than traditional machine learning using MRI texture features [18]. A feature extractor divides wrist X-rays into two categories based on the presence or absence of fractures. The most common method of target detection is divided into two stages and requires training of both models; the first stage identifies all suspicious areas that may contain regions of interest with high sensitivity and therefore a high rate of false positives.

The second stage is a simple classification of the subimages extracted in the previous step [19]. This method has been successfully applied to the detection of microbleeds in the brain with a sensitivity of 93% [20]. The second stage of the classification step is usually done by transfer learning. Although the application of deep learning in medical imaging is promising, there are some challenges and potential pitfalls. One of the main challenges is data availability, the data volume of medical images is usually much smaller, and biomedical data is usually unbalanced because the amount of data from normal sources is much larger than the amount of data from various abnormalities, and some studies have used data augmentation to increase the data volume to solve the data imbalance problem [21]. Secondly, the black-box nature of deep learning, even though the combination of deep learning and imaging has shown good performance, is still difficult to interpret in most cases. Is the technology acceptable in this era of evidence-based medicine? Therefore, deep learning is currently used as an adjunct rather than a replacement for the diagnostic work of radiologists. Third, research related to deep learning raises legal and ethical issues. No system can be perfect, but who will be responsible for the mistakes made by computers? As AI permeates all areas of human activity, such questions are likely to be researched and answered in the coming years. Finally, public acceptance is also something that should be considered in the development of deep learning [22].

In this study, a classical model of deep learning-based convolutional neural network (CNN), ResNet 50, was constructed and optimized. 18,152 mammographic images were collected from August 2015 to February 2018, and the mammographic density of the images was assessed by two experienced radiologists according to the ACR BI-RADS standard. Each fine-tuned classification model was evaluated for classification of breast density in a small dataset (4000 images) and in the original dataset (18152 images) to obtain the corresponding classification accuracy, and the classification performance of the model was classified as BI-RADS 4A, BI-RADS 3, and BI-RADS 2 for lesion assessment using the subject's working characteristic curve and area under the curve. The evaluation classification of lesions as BI-RADS 4B, BI-RADS 4C, and BI-RADS 5 was set to be inconsistent with the pathology control if the lesions were considered to have a low probability of malignancy, a high probability of malignancy, or a high suspicion of malignancy. Three comparison groups were used to evaluate the agreement between the classification and the pathological findings. The first group consisted of X-ray alone and ultrasonography; the second group consisted of X-ray alone and both tests in combination, and the third group consisted of ultrasonography alone and both tests in combination. The compliance rates of the three groups were compared using the x-test, and *P* value was <0.05. The differences between the two groups were statistically significant. The deep learning-based target detection algorithm can detect, localize, and classify the lesions on the mammography images with high accuracy, which provides radiologists with an auxiliary diagnosis for lesion identification and classification and makes a preliminary exploration for the further application of deep learning in medical image lesion detection.

## 2. Fully Digital Mammography Microtumour Classification Design

### 2.1. All-Digital Mammogram Analysis

A total of 18,152 images of 4549 patients (including 22 patients with unilateral mastectomy) who underwent all-digital mammography at our institution between August 2016 and December 2019 were retrospectively analysed, all of whom were females, with a mean age of 43 years, all of whom were normal or nonbreast cancer patients, and all of whom had no history of partial mastectomy or implantation. Breast density was assessed by two experienced radiologists in a double-blinded fashion according to the BI-RADS criteria established by the fifth edition of the ACR, and the results of the breast density assessment were recorded separately. Mammograms were obtained using a Hologic all-digital mammography machine, with both medial and lateral oblique (MLO) and cephalocaudal (CC) positions of both breasts (unilateral in postoperative patients) projected [23]. The deep learning-based breast classification model was built on the Porch framework with Ubuntu 18.04 operating system, running on two Titan 1080 graphics cards. The model was trained and tested on the Linux operating system.

FFDM images have a high resolution and good contrast, showing microcalcifications as small as 0.1 mm, allowing the observation of subtle changes in the lesion. The image postprocessing function can be adjusted through the window width and window position to obtain better contrast and brightness. The lesions can be measured, marked, etc. The images can be stored digitally, and remote consultation can be realized. FFDM can display the thicker structures in the centre of the breast, as well as the nipple, skin, and subcutaneous fat. The display of microcalcifications is much better than that of a traditional one-screen system, which improves the detection rate of breast cancer. In addition to the many advantages of FFDM in terms of image quality, the radiation dose of FFDM is 30–60% less than that of traditional mammography, which is still a great advantage over traditional one-screen mammography. Nowadays, FFDM is gradually replacing traditional screen-slice mammography, as shown in Figure 1. The mammograms of the 31 cases analysed in this review were supplemented with local compression photography combined with microlocal magnification in addition to the usual standard postural examination in each case. Compared with total breast compression, local compression plates are smaller than total compression plates, and local pressure is applied to the area of interest, resulting in a thinner local area of interest and better separation between the normal breast tissue and the lesion. The magnification is a small focal point of the X-ray bulb, usually 0.1 mm or less, and this comparative study uses a 0.1 mm small focal point magnification technique. The magnification can improve the display of lesion edges and more effectively show the number, shape, and distribution of calcification foci. Local compression photography combined with micrococcal magnification photography effectively improves the resolution of the images and the ability of distinguishing between benign and malignant lesions.

Before the completion of routine and adjunctive X-rays, a medical history is routinely completed, including the patient's chief complaint, as well as a history of childbirth, lactation, surgery, family history, and physical examination. To extract valid features, the tumour region is first segmented. In this paper, tumour segmentation of multimodal breast images is performed using a pretrained FCN network whose network architecture is adapted from the VGG16 network. The learning rate is fixed to IONA-IO; the momentum is set to 0.9, and the weight attenuation value is 0.0005. A loss function is constructed between the tumour regions manually delineated by experienced radiologists and the segmentation result map generated by the FCN network, and, by minimizing the loss function, the FCN network learns the tumour regions and the segmentation result map. The segmentation result map was as identical as possible to the manually delineated tumour regions. As the training process progressed, the tumour regions marked by the FCN network became closer and closer to the manually delineated tumour regions. After completing the training, the multimodal breast images were input into the pretrained FCN network, and the tumour regions were marked by heat maps as the segmentation results.

### 2.2. Classification Algorithm Analysis

Convolutional neural networks (CNNs), as the classical network for deep learning, have shown good classification performance in medical images, and they are highly adaptable and good at mining local features of data, extracting global features, and classifying them. A common CNN architecture is to stack several convolutional and rectification layers, add a pooling layer, and then use the full connection layer to control the output [24]. Different network models, such as LeNet, AlexNet, and ResNet, are built on top of this. The depth of the network is critical to the performance of the model. The increase in the number of network layers allows for more complex feature extraction, which in theory leads to better results; however, in practice, as the network depth increases, there is a network degradation problem, and the deep network has the problem of gradient disappearance or gradient explosion, making it difficult to train the deep learning model. The uniqueness of medical images requires network deepening, so we adopt a deeper network model based on CNN: ResNet 50 in the deep residual network (ResNet), as shown in Figure 2.

The model features a unique residual network block based on network deepening to solve the network performance degradation problem through constant mapping and reduce the number of parameters for computation. Therefore, using the ResNet 50 model can better train deeper CNNs and improve the accuracy of image classification and target detection. The loss function is a nonnegative real-valued function used to estimate the degree of inconsistency between the predicted value and the true value of the model, and the smaller the loss function, the better the robustness of the model. For the classification task of this study, a relatively good cross-entropy loss function is selected, and the following equation is the cross-entropy loss function formula:

(1) $$\begin{array}{c} C=-\frac{1}{n}\sum_{x}\left[y\;\ln\;a+\left(1-y\right)\log\left(1-a\right)\right]. \end{array}$$

Optimizer selection: an optimizer is used to update and compute the network parameters that affect model training and model output to approximate or reach the optimal value, thus minimizing the loss function; the best optimization method is the Adam optimization method, which is chosen for this paper. The main advantage of Adam is that the learning rate of each iteration has a defined range after bias correction, making the parameters smooth.

The traditional shape characteristics are too varied to be described in detail, so this article will focus on some common ones. Height to width ratio (HWR): if this ratio is greater than 1, it means that the nodule has a high probability of malignancy and requires attention.

(2) $$\begin{array}{c} \text{HWR}=\frac{\text{height}}{\text{width}}. \end{array}$$

The degree of roundness is determined by the ratio of the area of the nodule, *S*, to the circumference, *L* squared, reflecting the regularity in the shape of the nodule. The greater this value, the more irregular the shape of the nodule and the more likely it is to be malignant:

(3) $$\begin{array}{c} R=\frac{8\pi {}^{*}S^{2}}{3L^{2}}. \end{array}$$

MBR is the minimum external rectangular area, and tightness is positively related to the degree of nodule benignity:

(4) $$\begin{array}{c} S=\frac{S^{2}}{\text{MBR}}. \end{array}$$

The extraction process of texture features has a significant impact on the classification results. Currently, there are two main ways to extract texture features: one is the time-domain approach, where the grayscale values of the image pixels are counted and calculated, and then some texture features are generalized; the other is the use of frequency-domain correlation algorithm, which performs frequency-domain transformation or filtering to extract local texture features of the image through well-designed filters [25]. The ACR TI-RADS criterion reveals that malignant nodules usually have irregular image edges or even lobed edges that tend to extend outward toward the thyroid gland, and the internal structure is solid or almost completely solid, resulting in a strong echogenic calcification point on the image due to massive necrosis of the cells, whereas benign nodules have smooth edges and are generally spongy, cystic, or almost completely cystic inside because the internal structure is not smooth. There are no solids, mostly fluids, so there are no echoes and no calcification points. Therefore, properly designed texture features that effectively reflect these ultrasound sonographic features are of great importance for subsequent classification. Thus, the ACR TI-RADS criteria are also based on textural features, and, similarly, clinicians also observe the textural features of ultrasound images of nodules during the diagnostic process to make a benign or malignant determination.

The grayscale means value of the pixels of the ROI:

(5) $$\begin{array}{c} I_{\text{mean}}=\frac{\sum_{i=1}^{M}\sum_{j=1}^{N}I{\left(i,j\right)}^{2}}{M^{2}*N^{2}}. \end{array}$$

The grayscale variance of the pixels of the ROI:

(6) $$\begin{array}{c} I_{\mathrm{var}}=\frac{1}{n-1}\sum_{i=1}^{M}\sum_{j=1}^{N}I{\left(i,j\right)}^{2}. \end{array}$$

The grayscale standard deviation of the pixels of the ROI:

(7) $$\begin{array}{c} I_{\text{std}}=\sqrt{I{\left(i,j\right)}_{i}^{j}},\\ \text{Con}=\sum_{i}\sum_{j}{\left(i+j\right)}^{2}P{\left(i,j\right)}^{2},\\ \text{Corr}=\sum_{i}\sum_{j}\frac{{\left(i-u_{j}\right)}^{2}{\left(j-u_{i}\right)}^{2}}{\delta_{i}\delta_{j}},\\ \text{HGY}=\sum_{i,j=1}^{M}\frac{{\left(i-u_{j}\right)}^{2}{\left(j-u_{i}\right)}^{2}}{\chi_{i}\gamma_{j}}. \end{array}$$

To obtain features after convolution, the image is often minimally compressed, and upsampling (also known as deconvolution) is required to restore the original image. The two most popular approaches are deconvolution or bilinear interpolation. As shown in Figure 3, the FCN network has been pooled five times, the feature map size becomes 1/32 of the initial size, and the final convolution of the sixth and seventh layers does not change the size, only the number of features. At this point, the output feature map is called a heat map. After upsampling 32 times using the inverse convolution, the learning performance is better and the training is more efficient than bilinear interpolation.

After image cropping, data augmentation of the dataset is required. Data augmentation, also called data augmentation, refers to the ability of making a limited amount of data produce equal or more data value without substantially increasing the data. The best way to prevent model overfitting and to increase the generalizability of the model is to train large-scale datasets. In practice, however, acquiring clinical ultrasound images of uterine fibroids is very limited. Collecting patient data from a single outpatient clinic has a high time and economic cost and requires strong medical imaging experience in data annotation, making it difficult to accurately annotate on a large scale. This makes it difficult to train the model. Therefore, data augmentation was chosen to expand the existing dataset and add data copies, which is also a key to the success of this experiment.

By applying geometric or colour transformations and other graphical operations to the original images, data augmentation can obtain more data like the original data without changing the image feature information, making it easier for the model to obtain the invariant features of the training data. The following two points should be considered when amplifying the ultrasound images of uterine fibroids: the essential characteristics of the amplified dataset are consistent with the original data set, and the overall statistical characteristics of the dataset cannot be changed. The important clinical diagnostic features such as grayscale characteristics and texture information of the original lesion should be preserved in the amplified dataset. Therefore, in this paper, the geometric transformation was used to amplify the data, which maximizes the advantages of the dataset for network training in the case of limited training of the dataset.

## 3. Experimental Design Analysis

### 3.1. Experimental Design

8872 images of 2218 pathologically confirmed mammographic cases were annotated and classified by two radiologists using manual annotation software based on the histopathological findings and recorded by the two radiologists. All 2218 cases were divided into a training dataset of 1775 cases (80% of the total dataset) and a test dataset of 443 cases (20% of the total dataset). In the training phase, tenfold cross-validation was used, in the same way as in the first part, to optimize the model by continuously adjusting the parameters, and the mammogram images with manual annotation were entered.

The first target detection networks to be proposed were the region CNN (R-CNN) series, such as the VGG neural network, which eventually adopted an SVM classifier for classification. The greatest contribution of the R-CNN is selective search, which takes a segmentation approach to partition the image into small regions, using colour histograms. Rules such as the similarity of gradient histograms were merged, resulting in 2000 selection boxes. Given this, R-CNN has been greatly improved in speed and accuracy, and the subsequent Fast R-CNN integrates the idea of SPP-Net into R-CNNN, and its core contribution is that, firstly, the image first gets the feature layer through the neural network, and then the candidate frames generated by the selective search on the original image are mapped to the feature layer through the position, which avoids a large number of. The second is the use of Spatial Pyramid Pooling instead of the original pooling layer, so that there is no need to limit the size of the selection box. The most important contribution of the final Fast R-CNN is the use of regional proposal network (RPN), which enables end-to-end operation and shares the features of RPN and Fast R-CNN.

In the testing phase, the model's ability of localizing lesions and classifying them was verified by using a test dataset, in which mammographic images were input without any labeling, and the results were compared with the manually labelled lesions.

Statistical analysis was performed using MATLAB software. The evaluation indexes of the target detection model in this study were as follows: average precision (AP), mean average precision (mAP), and intersection-over-Union (IOU). Average precision (AP) is calculated from precision and recall; the higher the AP value, the better the classifier performance. The average precision (mAP) is the average of the APs for multiple categories. The mAP value evaluates the classification performance of the model on all categories. Intersection-over-Union (IOU), a concept used in target detection, is the ratio of the overlap between the selected candidate bound and the ground truth bound generated by target detection, i.e., the ratio of their intersection to their union. Therefore, in this study, IOU is used to evaluate the localization accuracy of target detection. The classification accuracy of the model was assessed using the subject's operating characteristic curve (ROC) and the area under the curve (AUC), and, in general, the larger the AUC, the better the relative performance of the model.

### 3.2. Indicator Design Analysis

The proposed breast tumour classification method is based on multimodal mammography and ultrasound data, i.e., a self-constructed dataset containing both mammography and ultrasound images of the same patient. To validate the necessity of multimodal fusion diagnosis, experimental comparison results between the correlation learning-based multimodal breast image classification (MCM) method and the unimodal breast image-based diagnostic method will be presented in this section. To make the comparison method experimental under the same conditions, the unimodal breast image-based diagnostic method consists of a unimodal data fitting term in the framework of this method and a regularized expression controlling the complexity of the single-optimal mapping matrix computation. The results of the experimental comparison of the performance of the MCM model with the unimodal breast image-based diagnostic method are presented in Figure 4, where *M* represents the results of the mammography-based breast tumour classification, and −*U* represents the results of the ultrasound-based breast tumour classification [25]. Also, to reduce the complexity of the original features and test the differences between different feature downscaling methods, five downscaling methods including LLE, MDS, IsoMax, SNE, and GPLVM were used in this paper to project the original high-dimensional features into the low-dimensional space of lower complexity, respectively. Despite the relatively small sample size of the dataset, a transfer learning approach is used in the experiment to migrate the training weight logs and parameters of the network's large-scale dataset and apply the training weights from the previous large-scale dataset to a new training session. With a relatively small amount of data, we can achieve good training results and avoid the problem of convergence when reinitializing the parametric model, thus improving the model segmentation accuracy.

Also, mammography is sensitive to calcified lesions and can determine the benign or malignant nature of the lesions by their shape, number, and distribution. Ductal carcinoma in situ, with microinfiltration, invasive ductal carcinoma, and inflammatory breast cancer are all characterized by small, polymorphic calcifications, but also by rough, inhomogeneous, and vague, indeterminate calcifications, with clusters, lines, and segments being the most typical distribution [26]. The calcification foci of nonspecific mastitis are coarser and larger than those of breast cancer and may appear as coarse rods or granules. The larger granular calcified plaques with translucent centres show “epithelial beading,” which is a specific calcification of plasma cell mastitis. Granulomatous mastitis has a lower incidence of calcification. The calcified foci of inflammatory breast cancer have the same characteristics as those of normal breast cancer; they are small and inhomogeneous. Foci of calcification are of moderate density and have irregular margins, while a few foci have large, smooth margins, like benign calcifications. Simple calcification is the most common form of ductal carcinoma in situ on X-ray, which is the main reason that an X-ray is more sensitive to the detection of ductal carcinoma in situ. Of the 31 cases of nonspecific mastitis analysed in this review, 2 cases showed coarse rod-shaped calcifications on mammography, and none showed any of the 4 manifestations of suspected malignant calcifications. Mammography can show the pattern and distribution of calcifications within the lesion in a way that mammography cannot compare with ultrasound.

## 4. Results Analysis

### 4.1. Analysis of Classification Results

In this study, as the number of iterations increased, the accuracy of the target detection model in classifying breast lesions as benign or malignant became stable, with 87% accuracy for benign lesions and 89% accuracy for malignant lesions. In this study, the target detection model classified the benign and malignant lesions in the test set as shown in Figure 5, in which there were 330 malignant lesions and 562 benign lesions in the test set, and 294 malignant lesions were correctly classified by the target detection model and 494 benign lesions were correctly classified by the target detection model. The accuracy rate was 89.2%, the precision rate was 81.2%, and the recall rate was 89.1%. Breast density, as one of the most important risk factors for breast cancer, can be used in breast cancer risk assessment prediction and surveillance and in determining individualized breast cancer screening protocols, but, at present, inconsistency in breast density assessment is a widespread problem. With the rise of deep learning, deep learning has shown good image recognition and classification ability in images without manual feature extraction, and its application in medicine is gradually increasing, and some scholars have introduced deep learning into the detection and diagnosis of breast diseases and even the study of breast pathological sections, but only a few studies have used deep learning for the measurement and classification of breast density. This is one of the factors that should be studied without delay.

The classification accuracy of the breast density classification model based on deep learning tends to stabilize as the number of iterations increases. When using the original dataset (18,152 images), the classification accuracy was 91% for category a, 89% for category b, 88% for category c, 90.75% for category d, and AUC of 0.9235 for category d. Compared with the small dataset, the classification accuracy for category d was 91.25% for category a, 89.45% for category b, 88.47% for category c, 90.58% for category d, and AUC of 0.9236. The AUC values of b and c are higher than those of the small dataset, indicating that the classification performance of the classification model gradually improves as the sample size increases, as shown in Figure 6.

The feature extraction process for qualitative breast density assessment in this study is particularly difficult, and the model constructed can directly simulate a radiologist making a visual assessment, but it is difficult to determine which specific part of the information is being simulated. This makes breast density classification more suitable for deep learning methods that do not require manual feature extraction. Therefore, a deep learning-based breast density classification model was first constructed that automatically classifies breast density by learning many images classified by radiologists. This method avoids the manual feature extraction process and is expected to achieve a more consistent breast density assessment, thus helping to improve the current qualitative breast density assessment and apply it in clinical practice, as shown in Figure 7.

From Figure 7, it can be seen that the AUC, accuracy, sensitivity, specificity, PPV, and NPV of the proposed MCM model are 95.83%, 95.00%, 91.67%, 95.83%, 95.83%, and 88.89%, respectively, which are slightly lower than those of the selectively integrated classifier in terms of sensitivity and NPV, probably because the source code is not available. Through the understanding and analysis of the method and experimental results, the method was reproduced using the dataset constructed in this paper with some differences. However, compared with existing classical classification methods, it achieves significant advantages in terms of AUC, accuracy, specificity, and PPV, etc., because the existing fusion classification methods usually use unimodal data to classify results. Also, the existing fusion classification methods usually utilize classification results based on unimodal data, independently generated from unimodal breast images; they ignore the relationship between multimodal breast images and suffer from the limitation of insufficient information from unimodal data. In contrast, by exploring the relationship between the two modalities, the MCM model proposed in this paper obtains more discriminatory information to jointly train the diagnostic model and achieve a more effective fusion. The experimental results in this subsection also demonstrate the superiority of the MCM model over the existing fusion classification methods.

### 4.2. Analysis of Experimental Results

Of the 136 malignant breast lesions, 28 cases (including 15 invasive ductal carcinomas, 7 intraductal carcinomas, 2 ductal carcinomas in situ, 2 mucinous carcinomas, 1 lobular carcinoma in situ, and 1 papillary carcinoma) were correctly diagnosed by digital breast tomography only, and 18 cases (including 10 invasive ductal carcinomas, 2 intraductal carcinomas, 1 papillary carcinoma, 1 mucinous carcinoma, 1 invasive lobular carcinoma, and 1 ductal carcinoma in situ) were correctly diagnosed by digital breast tomography only. Among the 128 benign lesions, 22 cases were overdiagnosed by digital breast tomography, 21 cases were overdiagnosed by ultrasound, and 11 cases were overdiagnosed by both digital breast tomography and ultrasound, as shown in Figure 8.

For the included lesions overall, the sensitivity and specificity of digital breast tomosynthesis were 86.03% (117/136) and 74.22% (95/128), respectively, for ultrasound, 78.68% (107/136) and 75.00% (96/128), and 94.12% (128/128), respectively, for combined diagnosis.

The sensitivity of digital breast tomosynthesis was higher than that of ultrasound and the specificity was slightly lower than that of ultrasound, and the differences were not statistically significant (*P* > 0.05). The sensitivity of the combined diagnosis was higher than that of digital breast tomosynthesis and ultrasound (*P* < 0.05), and the specificity was higher than that of digital breast tomosynthesis and ultrasound (*P* > 0.05). The ROC curves of digital breast tomosynthesis, ultrasound, and combined diagnosis are shown in Figure 9, with the lower areas of 0.801, 0.768, and 0.869, respectively. The difference between combined diagnosis and digital breast tomosynthesis or ultrasound on the lower area of the ROC curve of the overall lesion was statistically significant (*P* < 0.05), while the difference between digital breast tomosynthesis and ultrasound on the lower area of the ROC curve was not statistically significant (*P* > 0.05).

As a comparison, three separate classifiers for the three feature channels were designed in this paper, three ResNet models were used to compare with our integrated learning model, and comparative experiments were conducted on the four-classification metrics of the models. The results of the three separate classification models and our integrated learning model are shown in Figure 10. The accuracy, sensitivity, specificity, and AUC area of our model are significantly higher than those of the other three separate models, which proves that the overall performance of our model is better.

Among the target detection models, this study introduces its most important evaluation metric, mAP value, which evaluates the classification performance of the model on all categories and provides a more intuitive and objective evaluation of the model's classification performance. Combining the target detection model with the ResNet network model, which was optimized in the first section, makes it more suitable for medical images. We need to further expand the data volume to include more imaging signs to further improve the classification of benign and malignant tumours of the breast and secondly include more histopathologically confirmed breast cancer cases. The target detection model has been widely used in histological classification of breast cancer. The convolutional neural network model ResNet 50 was used for the breast density classification task. Methodological innovation: the data used in the study directly adopts the real data from hospitals, which truly reflects the individual differences in breast images; the age group of the examined patients is concentrated, and the data of categories b and c are larger, which also reflects the distribution of breast density; the breast density is classified into four categories according to BI-RADS, which is in line with the routine clinical diagnosis. A related study showed that the correlation between breast density and breast cancer risk was not found after classifying breast density into fatty and dense types, but it was found to be correlated with breast cancer risk after classifying breast density into four categories according to BI-RADS criteria. Therefore, the four categories according to the BI-RADS criteria in this study are clinically meaningful.

## 5. Conclusion

To improve the accuracy of detection and diagnosis of breast lesions on mammography images, this study builds a deep learning-based target detection model for breast X-ray lesions and initially discusses the value of a deep learning-based target detection algorithm in detecting, localizing, and classifying breast lesions in full digital mammography examinations. The target detection model has an IOU of 87% for localization accuracy, 89.1% for classification sensitivity, 87.9% for specificity, and 89.2% for classification performance AUC. The mAP value of 90.4% indicates that the target detection model has good classification performance for benign and malignant mammary lesions. In this paper, we present the results of the first partitioning model, Mask RCNN, in which the ResNet structure is used to extract features efficiently, and the RPN network is combined with the RPN network to achieve feature and efficient utilization and fusion. The accuracy of 84.76% and 87.05% was achieved, which proved the accuracy and feasibility of the two models. The practical value of the deep learning image segmentation method for evaluating HIFU ablation efficacy was demonstrated. The average absolute percentage error was 14.8%, which verified the practical value of the model from the perspective of clinical application and achieved the cross-application of deep learning and medical image segmentation.

## Figures and Tables

**Figure 1:** All-digital mammogram.

**Figure 2:** Classification algorithm framework.

**Figure 3:** Experimental design steps.

**Figure 4:** Performance specification design.

**Figure 5:** Classification of the test set foci by target detection model.

**Figure 6:** ROC curves of the classification performance of the model for different data sets for breast density.

**Figure 7:** Performance comparison of classification methods.

**Figure 8:** Example of experimental results.

**Figure 9:** ROC curves for DBT, ultrasound, and combined diagnosis of total lesions.

**Figure 10:** Comparison of the effects of different classification models.

## Data Availability

The data used to support the findings of this study are available from the corresponding author upon request.
